The article "Multiclass Cancer Prediction Based on Copy Number Variation Using Deep Learning" was published in 2022. Journal: Comput Intell Neurosci.

# Multiclass Cancer Prediction Based on Copy Number Variation Using Deep Learning

**DOI:** 10.1155/2022/4742986

**Published:** 2022-06-09

**Authors:** Haleema Attique, Sajid Shah, Saima Jabeen, Fiaz Gul Khan, Ahmad Khan, Mohammed ELAffendi

**Affiliations:** ^1^Department of Computer Science, COMSATS University Islamabad, Abbottabad Campus, Islamabad, Pakistan; ^2^EIAS Data Science Lab, College of Computer and Information Sciences, Prince Sultan University, Riyadh, Saudi Arabia; ^3^Department of IT and Computer Science, Pak-Austria Facchochschule: Institute of Applied Sciences and Technology, Mang, Haripur, KPK, Pakistan

## Abstract

DNA copy number variation (CNV) is the type of DNA variation which is associated with various human diseases. CNV ranges in size from 1 kilobase to several megabases on a chromosome. Most of the computational research for cancer classification is traditional machine learning based, which relies on handcrafted extraction and selection of features. To the best of our knowledge, the deep learning-based research also uses the step of feature extraction and selection. To understand the difference between multiple human cancers, we developed three end-to-end deep learning models, i.e., DNN (fully connected), CNN (convolution neural network), and RNN (recurrent neural network), to classify six cancer types using the CNV data of 24,174 genes. The strength of an end-to-end deep learning model lies in representation learning (automatic feature extraction). The purpose of proposing more than one model is to find which architecture among them performs better for CNV data. Our best model achieved 92% accuracy with an ROC of 0.99, and we compared the performances of our proposed models with state-of-the-art techniques. Our models have outperformed the state-of-the-art techniques in terms of accuracy, precision, and ROC. In the future, we aim to work on other types of cancers as well.

## 1. Introduction 

The change in the DNA refers to the term genetic variation which makes us all unique. There are different forms of genetic variation, and most of them are well understood. It can involve changes in the DNA nucleotide or chromosome structure [1, 2]. Human genome is well-off in structural variation where copy number variation (CNV) is the most communal type which is the change in the number of copies in a specific area of the genome [3]. In the 1000 Genome Project data, CNV is known as copy number polymorphism (CNP) [4]. CNVs are DNA regions ranging in size from 1k bases to several megabases [5]. CNV is normally due to insertion, deletion, and/or duplication of the chemical bases (nucleotides). Some CNVs appear first time in the parent's germ cell called de novo, while others are inherited [6]. Usually, the cell has two copies of each gene; CNV occurs when a part of a gene is deleted or duplicated [7].

The article "Multiclass Cancer Prediction Based on Copy Number Variation Using Deep Learning" was published in 2022. Journal: Comput Intell Neurosci.

Copy number variations affect transcription in humans [8] and have been related to different diseases such as cancer, autism, and schizophrenia [9–11]. All over the world, the most common risk that impends human health is cancer [12]. Cancer is a class of disease which results in irregular growth of cells and is one of the leading causes of human death. The mortality rate of humans due to cancer is about 14.6% each year [13]. Phenotypic variation may also be due to CNVs [6, 14]. The data obtained from CNVs can also be used to classify tumors into malignant and benign [15, 16]. A number of research articles agree that somatic CNVs are mostly associated with the progression of various cancers [17–20].

Machine learning practitioners have proposed a lot of techniques to identify one or multiple types of cancer(s) using various types of genomic data, each with different weaknesses and strengths. During the health checkup, the colonoscopy screening is broadly known for the evaluation of colorectal cancer (CRC) risk, but due to its discomfort and complexity, more reliable and comfortable methods were necessary for the CRC screening. A comprehensive study is presented by Ding et al. [21] about machine learning applications in CNV-based cancer prediction.

Dealing with high-dimensional and heterogeneous data remains a key challenge in healthcare [22]. Traditional methods of machine learning firstly need to perform feature extraction and selection to obtain more useful features from the data and then build prediction models on them. The advancement in deep learning technologies provides effective approaches to obtain end-to-end learning models. Deep learning is a fashionable toolbox and has become popular for big data [23, 24] especially in the field of genomics due to its performance in prediction problems. It is used for many processes such as predicting DNA sequence conversation, identifying enhancers and promoters, and detecting genetic variation from DNA sequencing. The advancement and fruitful applications of deep learning in different fields of genomics reveal that it can be used for cancer classification from CNV data [22, 25–27].

Different computational models for the cancer classification based on copy number variation data are available. The most recently developed model achieves an accuracy up to 85%. The copy number variation data are high dimensional in nature and difficult to handle by the classical machine learning techniques. In this study, we implemented deep learning models that successfully used 24,174 genes of CNV levels to classify six types of cancers: breast adenocarcinoma (BRCA), urothelial bladder carcinoma (BLCA), colon and rectal carcinoma (COAD/READ), glioblastoma multiforme (GBM), kidney renal clear cell carcinoma (KIRC), and head and neck squamous cell (HNSC). The highest obtained average training accuracy is 96%, while testing accuracy is 92%. We have proposed three different deep learning architectures, and all of these models have outperformed state-of-the-art techniques in terms of accuracy, ROC, and precision, while two of our networks have outperformed the state-of-the-art models in terms of recall (see Table 1). So, the contribution of this work is not only to improve the performance (accuracy) of the cancer classifier using an end-to-end model but also to find out which architecture among DNN (deep fully connected neural network), CNN, and RNN is suitable for CNV data. According to our finding, DNN performs better than the rest of the two.

The article "Multiclass Cancer Prediction Based on Copy Number Variation Using Deep Learning" was published in 2022. Journal: Comput Intell Neurosci.

We have discussed the literature review in Section 2, while Section 3 covers the explanation of the dataset and architectures of our models.  Section 4 deals with the training process of our models along with obtained results and our findings. Finally, we have concluded our work in Section 5.

## 2. Related Work

Xu et al. [28] have identified the chromosomal alterations in plasma for early detection of CRC. They analyzed the CNVs in cfDNA (cell-free DNA) by using the regular *z* score, and the SVM classifier was trained for identification of colon and rectal cancers. The patients with early two stages (I and II) were detected. Brody et al. [29] used blood samples of 8,821 different patients. For feature extraction, they have extracted germline DNA copy number variation data by a single laboratory with an SNP 6.0 array. The gradient boosting algorithm is used to predict breast, ovarian, brain, and colon cancers. Ricatto et al. [30] used a discretizer for feature extraction and a fuzzy rule-based predictor for tumor classification.

In women, breast cancer is the most common type of cancer, which has further subtypes [31]. Pan et al. [32] carried out feature extraction and selection using MCFS (Monte Carlo feature selection). IFS (incremental feature selection) is used to better represent the core CNVs in different subtypes of breast cancer, and then, the dag-stacking model is integrated to detect multiple types of breast cancer. Islam et al. [33] focused on the prediction of molecular subtypes of breast cancer. They performed the experiments to identify binary classes, i.e., estrogen receptor (ER+ and ER−) and multiple classes, i.e., PAM50 (luminal A, luminal B, Her2 enriched, and basal-like). Afterwards, they performed the chi-square test to select the topmost significant genes. For classification, DCNN (deep convolution neural network) was used. Lu et al. [34] also focused on the classification of breast cancer. The authors have introduced a module-based network integrated with genomic data to identify important driver genes in BRCA subtypes. CNV analysis was performed by Li et al. [35] on tumor development. The use case was breast cancer, where they collected data from the TCGA-BRCA project. They searched OMIM (Online Mendelian Inheritance in Man) for most relevant CNVs. They have chosen six candidate genes: ErbB2, AKT2, KRAS, PIK3CA, PTEN, and CCNDI. Furthermore, they have constructed two types of distance-based oncogenetic trees to find which of the above candidate genes play a significant role in the development of breast cancer. Their findings showed that ErB2 has early alteration, while AKT2, KRAS, PIK3CA, PTEN, and CCNDI have late alterations in human breast cancer. Alshibli et al. [36] have proposed deep convolution-based neural networks for CNV data to classify six types of cancer. They have lent the famous computer vision architectures, i.e., ResNet16 and VGG16. Their average accuracy is 86%. They reported that their proposed model has the lowest performance for UCEC (uterine corpus endometrial carcinoma).

The article "Multiclass Cancer Prediction Based on Copy Number Variation Using Deep Learning" was published in 2022. Journal: Comput Intell Neurosci.

To understand the association of CNVs with various types of human cancer, Zhang et al. [37] collected CNV data of different cancer classes consisting of 24,174 genes as features. The feature selection was carried out using minimal redundancy maximal relevance (mRmR) and incremental feature selection (IFS), which resulted in the selection of 200 genes. The dagging model is used for the classification phase of multiple types of cancer. Fekry et al. [38] also worked on these CNV levels of 24,174 genes to classify a set of human cancer types named as breast adenocarcinoma (BRCA), urothelial carcinoma (BLCA), colon and rectal carcinoma (COAD/READ), glioblastoma multiforme (GBM), kidney renal clear cell carcinoma (KIRC), and head and neck squamous cell (HNSC). They selected 16,381 important genes of CNV levels using the filter method (i.e., information gain). For classification, they used seven different classifiers: support vector machine, j48, neural network, random forest, logistic regression, dagging, and bagging. The authors in [39] have contributed to cancer classification using the self-normalizing neural network. They have used Monte Carlo feature selection and incremental feature selection (IFS). They have worked on multiple cancer types and obtained 79% accuracy.

Most recently, researchers are using CNV data along with other modalities such as clinical and/or gene expression data to improve the performance metrics of their models. A contribution is made by researchers in [40] using multimodality data to classify subtypes of breast cancer with the help of the SVM (support vector machine) and RF (random forest). A deep learning model using multi- modality data is used to predict the subtype of breast cancer in [41, 42]. Another deep learning model along with multimodalities of data is used in [43] to predict Alzheimer's disease. The researchers in [44] have trained their deep learning model on multimodalities to predict therapeutic targets in breast cancer. A comprehensive comparison of multimodalities is presented in [45].

The article "Multiclass Cancer Prediction Based on Copy Number Variation Using Deep Learning" was published in 2022. Journal: Comput Intell Neurosci.

## 3. Materials and Methods

### 3.1. Dataset

For experimentation, we have selected the same dataset used by [38] in order to be compatible in result comparison. The said dataset is composed of six cancer types containing DNA CNVs of 24,174 genes (features/dimensions) for 2916 samples; therefore, the shape of the dataset is *X*_2916×24174_ if *X* is the input dataset. This dataset was taken from the cBioPortal for Cancer Genomics database http://cbio.mskcc.org/cancergenomics/pancan_tcga/. The database contains 11 different types of cancer, and each cancer type has its own samples. The CNV levels were regularized into five distinct values in the database with −2 for homozygous deletion, −1 for heterozygous deletion, 0 for diploid, 1 for low-level gain, and 2 for high-level gain. In this research, we used six different types of cancer, which are listed in Table 2, with names and the number of samples in each class (cancer type).

### 3.2. Our Proposed Models

#### 3.2.1. DNN (Deep Fully Connected Neural Network)

An artificial neural network (ANN) is a powerful computational tool that mimics the human brain working behavior [46]. A neural network (NN) consists of a set of neurons arranged in layers such as the input, hidden, and output layer. A single neuron takes an input vector, calculates the weighted sum, and applies the activation function to decide whether it should fire or not. In the fully connected neural network, every neuron of the previous layer is connected to all neurons of the next layer.

For a network of *L* number of layers, the *l*^th^ layer is specified by the associated weight matrix *W*^[*l*]^ ∈ *ℜ*^*n*^[*l* − 1]^×*n*^[*l*]^^, where *n*^[*l* − 1]^ and *n*^[*l*]^ represent the number of neurons in previous and current layers, respectively. The weighted summation of the *l*^th^ layer is given by

(1) $$\begin{array}{c} Z^{\left[l\right]}=W^{T}A^{\left[l-1\right]}+b^{\left[l\right]}, \end{array}$$

where *b* ∈ *ℜ*^*n*^[*l*]^×1^ is the bias vector and *A*^[*l* − 1]^ ∈ *ℜ*^[*l* − 1]×1^ is the activation map of the previous layer.

The article "Multiclass Cancer Prediction Based on Copy Number Variation Using Deep Learning" was published in 2022. Journal: Comput Intell Neurosci.

To speed up the network convergence [47], we have used the batch normalization that scales the *Z*^[*l*]^ in a specified range.  Algorithm 1 explains the batch normalization in detail.

In Algorithm 1, the parameters *γ* and *β* maintain the expressive power of the network, while *ϵ* is a small positive constant added for computational stability [48]. During the forward pass, an activation map *A*^[*l*]^ is estimated for each layer, *l*=1,2,…*L*, to know which neuron should be fired:

(2) $$\begin{array}{c} A^{\left[l\right]}=g\left({\tilde{Z}}^{\left[l\right]}\right), \end{array}$$

where *g* is the activation function. Here, we have used the rectified linear unit (ReLU) as an activation function for all hidden layers:

(3) Al=ReLUZ˜l=max0,Z˜l.

The ReLU expedites the training and avoids the vanishing gradient [49]. The last layer in the network is called the output layer (classification layer), which gives the probability of occurrence of different classes. Let there are *K* classes, and then, the probability of the dominant class is given by the softmax function:

(4) $$\begin{array}{c} \hat{y}=\underset{k}{\arg\;\max}\left\{\frac{e^{z_{k}^{\left[L\right]}}}{\sum_{k=1}^{K}e^{z_{k}^{\left[L\right]}}}\right\}, \end{array}$$

where *z*_*k*_^[*L*]^ is the weighted sum of the *k*^th^ unit of output layer *L*. In our case, the data contain six classes; thus, we set *K*=6.

In the deep fully connected neural network (DNN) category, we have implemented the networks from shallow to deep by increasing hidden layers one by one. Furthermore, the number of neurons is reduced with a factor of∼2 from beginning to end, to achieve dimensionality reduction. We started with a network of three hidden layers as shown in Figure 1 and continued up to seven layers. Aforementioned, we have used ReLU as an activation function in hidden layers with batch normalization and softmax at the output layer. To overcome the issue of overfitting, we have used dropout layers as well. For more details about the dropout layer, read the work of Srivastava et al. [50]. Note that, each input vector *X* contain 24,174 features, while the activation map, *A*^[*L* − 1]^, of the last hidden layer contains 150 features, which shows dimensionality reduction. For training, the Adam optimization algorithm along with categorical crossentropy as a loss function is used.

#### 3.2.2. 1D Convolutional Neural Network

We have also used the 1D1  *D* convolutional neural network (1D − CNN) for cancer classification. Normally, the CNN contains two parts: (1) convolutional layers that are responsible for feature extraction [51, 52] and(2) the fully connected layer that is responsible for classification. Our proposed 1D − CNN contains two convolutional layers followed by one fully connected layer. Every convolution layer is followed by a stack of max pooling, batch normalization, and dropout layers.  Figure 2 presents the detailed architecture of the proposed model.

The article "Multiclass Cancer Prediction Based on Copy Number Variation Using Deep Learning" was published in 2022. Journal: Comput Intell Neurosci.

Note that, the first convolutional layer contains 20 filters, each of size 5, and the ReLU as an activation function. Similarly, the second convolutional layer consists of a stack of 10 filters, each of size 5, and the ReLU as an activation function. For the activation function in the output layer, we have used softmax (See equation (4)).

#### 3.2.3. LSTM (Long Short-Term Memory)

LSTM is one of the popular flavors of the RNN (recurrent neural network) with three special gates, i.e., the input/update, forget, and output gate, as shown in Figure 3. The key gate is the forget gate that is used to keep long-term dependency intake. It is the long-term dependency preservation that makes LSTM suitable for sequential data analysis [53].

In our proposed model, we have used 24 LSTM units, ReLU as an activation function followed by a batch normalization layer and then the output layer.

## 4. Results and Discussion

The dataset was split into training and testing with 80% and 20%, respectively, to examine the performance of our proposed models. The methodology that we have adopted is shown in Figure 4. The testing and validation dataset are the same; that is why, validation and testing metrics are the same. The representation learning implicitly exists in the model (s). The worth of representation learning using deep learning has been proved in the literature. As mentioned in Section 3.2, we have implemented three different neural network architectures, to explore their strengths and weaknesses. We have started from the shallow neural network to the deep NN (deep fully connected NN), to LSTM to the 1D-CNN.

We have trained our models up to 200 epochs and plotted the results to check the training status, that is, to find whether the model is underfitted, overfitted, or properly trained.

The obtained training vs. validation accuracies of each model are shown in Figure 5. Given the results in Figure 5 our shallow NN (DNN_3_) and 1D-CNN require more epochs for training, while the remaining deep architectures require less epochs to reach the point where the model starts overfitting. The sign of overfitting is that when the training accuracy improves, while the validation accuracy starts to decline or remains the same. The possible reason behind this behavior is that the deep architecture normally extracts complex but well representative features.

The article "Multiclass Cancer Prediction Based on Copy Number Variation Using Deep Learning" was published in 2022. Journal: Comput Intell Neurosci.

A classwise ROC is shown in Figure 6. The highest ROC, i.e., 1.0 is achieved by all networks for the COAD/READ class, while the average maximum ROC is 0.99 achieved by NN_3_ (deep fully connected neural network with 3 layers) and DNN_5_ (NN with 5 layers) as shown in Table 1.

In order to test the performance of our networks for each class (cancer type), we have presented the computed results in Table 3. According to the obtained results, the GBM class is the most complex (difficult) one for our networks, while COAD is the easiest one. The same results can be verified from the confusion matrices given in Tables 4–5.

The average performance measures (in terms of accuracy, precision, recall, and ROC) of all networks are shown in the first four rows of Table 1. The obtained results show that our DNN architecture has outperformed the rest of our models.

We have compared our computed results with the state-of-the-art models. As mentioned in Table 1, our all networks have outperformed all of our competitors in most of the performance metrics. We have reported only the best results of Sana et al. [38]. Their maximum accuracy is 85% with an ROC area of 0.96, whereas our proposed models achieved the accuracy over 92% with an ROC of 0.99.

Since Zhang et al. [37] have worked similarly, but their research deals with some different types of cancers, e.g., UCEC (uterine corpus endometrial carcinoma); therefore, the comparison is not compatible, but they have achieved 75.1% accuracy.

In the light of the analysis made on the obtained results, we conclude that due to the small size of the current dataset, very deep neural networks are not beneficial to use as most of our models are converged with the small number of hidden layers. Moreover, the fully connected neural network performed better than other flavors such as CNN and RNN for copy number variation (CNV) data (see Table 1). We also found that adding additional layers to a fully connected neural network (DNN) has a small impact on results. Our obtained results also verify that end-to-end deep learning models are better in representation learning than handcrafted feature extraction (see Table 1)

## 5. Conclusion and Future Directions

Copy number variations are related to different human diseases, such as cancer, autism, and schizophrenia. In this paper, we classified six different types of cancers by using copy number variation data. We have proposed three different neural network architectures to make the classification process end-to-end. Moreover, we have effectively used the data-hungry nature of the deep neural network and we have not used the feature engineering (handcrafted feature extraction) step as used by most of the researchers to save computational time. Our achieved testing accuracies are 91%, 92%, 90%, and 91% by using CNV levels of 24,174 genes. Our work testifies that the CNVs of these genes play a crucial role in classifying human cancers. In the future, we aim to work on the other types of cancer as well.

The article "Multiclass Cancer Prediction Based on Copy Number Variation Using Deep Learning" was published in 2022. Journal: Comput Intell Neurosci.

## Figures and Tables

**Figure 1:** The architecture of the fully connected model with three hidden layers.

**Figure 2:** 1D convolution-based architecture.

**Figure 3:** LSTM architecture.

**Figure 4:** Our methodology.

**Figure 5:** Classification of accuracy of different models: (a) DNN_3,_ (b) DNN_5,_ (c) LSTM, and (d) 1D-CNN.

**Figure 6:** ROC of different models on various cancer types: (a) DNN_5,_ (b) LSTM, and (c) 1D-CNN.

**Algorithm 1:** Batch normalization.

**Table 1:** The average performances of different models along with the state of the art.

S. no	Models	Train Acc	Val Acc (%)	ROC area	Precision	Recall
1	DNN_3_	95%	91	0.99	0.88	0.87
2	DNN_5_	96%	**92**	0.99	0.89	0.88
3	LSTM	95%	91	0.98	0.89	0.85
4	1D-CNN	88%	90	0.98	0.88	0.85
5	Sana Fekry et al. [38]	—	85.9	0.965	0.852	0.862

**Table 2:** The distribution of samples with respect to each cancer type in our dataset.

Sr.	Cancer type	No of samples
0	BRCA (breast carcinoma)	847
1	BLCA (bladder urothelial)	135
2	COAD/READ (colon and rectal adenocarcinoma)	575
3	GBM (glioblastoma multiforme)	563
4	KIRC (kidney renal cell carcinoma)	306
5	HNSC (head and neck squamous cell)	490
Total		2916

**Table 3:** The classwise performances of all networks.

Models	GBM (3)	KIRC(4)	HNSC(5)	COAD/READ(2)	BLCA(1)	BRCA(0)
NN						
TP rate	0.68	0.96	0.82	0.98	0.83	0.93
ROC area	0.97	0.99	0.97	1.00	0.98	0.99
Precision	0.77	0.90	0.92	0.93	0.81	0.97
*F*-measure	0.72	0.93	0.87	0.96	0.82	0.95
Recall	0.68	0.96	0.82	0.98	0.83	0.93
FP rate	0.00	0.01	0.04	0.01	0.02	0.00

DNN						
TP rate	0.72	0.96	0.85	0.98	0.85	0.94
ROC area	0.97	0.98	0.99	1.00	0.98	0.99
Precision	0.75	0.93	0.94	0.94	0.85	0.93
*F*-measure	0.73	0.94	0.89	0.96	0.85	0.94
Recall	0.72	0.96	0.85	0.98	0.85	0.94
FP rate	0.01	0.02	0.01	0.01	0.01	0.01

LSTM						
TP rate	0.52	0.95	0.85	0.98	0.88	0.92
ROC area	0.96	0.99	0.98	1.00	0.97	1.00
Precision	0.87	0.91	0.93	0.92	0.79	0.95
*F*-measure	0.65	0.93	0.88	0.95	0.83	0.94
Recall	0.68	0.94	0.84	0.96	0.79	0.91
FP rate	0.52	0.95	0.85	0.98	0.88	0.92

1D-CNN						
TP rate	0.64	0.93	0.92	0.96	0.77	0.91
ROC area	0.97	0.99	0.97	1.00	0.97	0.99
Precision	0.84	0.93	0.81	0.93	0.86	0.94
*F*-measure	0.73	0.93	0.86	0.94	0.82	0.92
Recall	0.64	0.93	0.92	0.96	0.77	0.91
FP rate	0.00	0.02	0.04	0.01	0.01	0.01

**Table 4:** Confusion matrix for training data.

	BRCA(0)	BLCA(1)	COAD/READ(2)	GBM (3)	KIRC(4)	HNSC(5)
BRCA(0)	**109**	0	1	0	0	0
BLCA(1)	0	**673**	6	0	0	0
COAD/READ(2)	0	1	**470**	0	0	0
GBM (3)	0	0	2	**446**	0	0
KIRC(4)	0	0	7	0	**233**	0
HNSC(5)	0	0	3	0	0	**381**

The article "Multiclass Cancer Prediction Based on Copy Number Variation Using Deep Learning" was published in 2022. Journal: Comput Intell Neurosci.

**Table 5:** The confusion matrix for testing data.

	BRCA(0)	BLCA(1)	COAD/READ(2)	GBM (3)	KIRC(4)	HNSC(5)
BRCA(0)	**15**	1	2	2	3	2
BLCA(1)	0	**158**	3	3	2	2
COAD/READ(2)	0	3	**94**	1	4	2
GBM (3)	0	0	1	**113**	1	0
KIRC(4)	1	5	1	0	**55**	4
HNSC(5)	1	0	3	1	1	**100**

## Data Availability

The data are publicly available at this link: http://cbio.mskcc.org/cancergenomics/pancan_tcga.
